# Triumvirate Presentation and Treatment of Psoriasis in the Setting of HIV and Treponema pallidum Infection

**DOI:** 10.7759/cureus.22129

**Published:** 2022-02-11

**Authors:** Ariel Kidron, Hiep Nguyen, Hoang Nguyen

**Affiliations:** 1 Emergency Medicine, Nova Southeastern University Dr. Kiran C. Patel College of Osteopathic Medicine, Fort Lauderdale, USA; 2 Orthopaedic Surgery, Nova Southeastern University Dr. Kiran C. Patel College of Osteopathic Medicine, Fort Lauderdale, USA; 3 Basic Sciences, Nova Southeastern University Dr. Kiran C. Patel College of Osteopathic Medicine, Clearwater, USA

**Keywords:** human immunodeficiency virus (hiv) infection, hiv dermatoses, management of psoriasis, cutaneous syphilis, psoriasis pathophysiology

## Abstract

Psoriasis is an autoimmune condition in which the immune system attacks healthy skin cells, causing the accelerated formation of new skin characterized by scaly patches or plaques. These lesions are formed due to the formation of new skin underneath dead skin that has yet to be shed. Although the cause of psoriasis is not completely understood, it has been associated with infections that may trigger or exacerbate the condition. Syphilis, a highly infectious sexually transmitted disease, may trigger a psoriasis outbreak; because syphilis is known as “the great imitator”, it can present as many other chronic dermatoses and therefore often makes it very difficult to diagnose. Here, we describe a case of a 17-year-old Vietnamese male from Dong Nai Province who was initially diagnosed with psoriasis and later diagnosed with syphilis and HIV infection upon further investigation and testing.

## Introduction

Psoriasis is an inflammatory condition characterized by sharply demarcated, erythematous, scaly, pruritic plaques. It can develop in the setting of the human immunodeficiency virus (HIV) infection and may provide clinical signs of the degree of infection [1]. Psoriasis may also be mimicked by infection of *Treponema pallidum* causing destruction of the vasa vasorum of blood vessels and manifesting as an inflammatory rash [2]. Owing to the location the patient presented in Ho Chi Minh city, endemic syphilis is a likely causative factor, and this duality may present challenges to clinicians in successful diagnosis and treatment. Psoriasis is prevalent in 2% of HIV patients with an atypical, resistant, and more severe presentation of symptoms than the general population [3]. Here, we present a case of a 17-year-old Vietnamese male from Dong Nai Province who was initially diagnosed with psoriasis and later diagnosed with syphilis and HIV infection, thus presenting a triumvirate relationship between infectious and immunogenic etiologies to draw attention to the mimicking ability of syphilis, the coexisting nature of autoimmune and infectious diseases, and the differential diagnosis of cutaneous palmoplantar lesions.

## Case presentation

A 17-year-old Vietnamese male presented to a Dermatology Specialist Hospital in Ho Chi Minh City, Vietnam, with a chief complaint of red, scaly skin. Physical examination revealed erythematous plaques distributed on the ankles and body and lichenification on the back. He was initially diagnosed with psoriasis and treated with a course of 0.1% topical triamcinolone. The patient was subsequently admitted upon reevaluation following two months, where the clinical examination of his skin revealed 1-3 cm erythematous and violaceous plaques with central scales distributed on the neck, back, and extremities known as "target lesions." The densely distributed plaques on the distal extremities were coalescent and xerotic (Figure 1).

**Figure 1:** Skin examination revealed 1-3 cm erythematous and violaceous plaques with scaled centers (black arrow) on the neck, nipples, lower abdomen, umbilicus, lower extremities, upper extremities, and back.

A complete blood count revealed 12.49% monocytes (normal value is 0%-12.0%), 0.93 x 103/mm^3^ lymphocytes (normal value is 1.0-3.0 x 103/mm^3^), and 0.9 x 103/mm^3^ monocytes (normal value is 0.2-0.8 x 103/mm^3^). The patient was started on Augmentin 2g/day, acitretin 50g/day, vitamin E 4,000IU/day, chlorpheniramine 4mg/day, and zinc 20mg/day, and salicylic acid 5%, eosin 2%, and Daivobet were applied topically daily for suspected psoriasis. Skin biopsies from the back and leg revealed hyperplasia of stratum spinosum and stratum corneum with Munro-Saboureau microabscesses beneath the corneum and chronic inflammatory infiltrate with a vascular proliferation of the dermal papillae (Figure 2). Pathology confirmed a diagnosis of psoriasis with a superinfection. An additional skin biopsy of the patient’s right ankle exhibited stratum spinosum and corneum hyperplasia, spongiosis, numerous neutrophils, and plasma cell infiltration of the epidermis (Figure 3).

**Figure 2:** Histopathological findings. Histopathological findings of the lesions revealed hyperplasia of stratum spinosum and corneum with Munro-Saboureau microabscesses beneath the corneum and chronic inflammatory infiltrate with vascular proliferation of dermal papillae. Magnification, x10. Hematoxylin and eosin stain.

**Figure 3:** Histopathological findings. Histopathological findings of 0.5 x 1 cm right ankle skin lesion biopsy specimen revealed stratum spinosum and corneum hyperplasia, spongiosis, numerous neutrophils, and plasma cell infiltration of the epidermis. Magnification, x40, and x400, respectively. Hematoxylin and eosin stain.

The immunofluorescence assay of the ankle skin specimen was negative for IgG, IgA, IgM, fibrinogen, and C3. The skin lesions did not significantly improve with initial treatment, and thick, brown scales formed on his feet and ankles. Following biopsy results, *Treponema pallidum* rapid plasma reagent (RPR), *Treponema pallidum* hemagglutination assay (TPHA), and a rapid HIV antibody blood test were performed. The RPR was reactive in 512 dilution (R-512), signifying a positive screen, and TPHA was positive +++, confirming a syphilis diagnosis. The rapid HIV antibody test was also positive. One dose of benzathine penicillin G 2.4 million units intramuscularly (IM) was administered, and acitretin, vitamin E, chlorpheniramine, salicylic acid 5%, and Daivobet were continued for 12 more days. All other medications were discontinued. The erythema and the scaly plaques significantly decreased, and skin exposure improved. The patient was discharged and referred to an infectious disease specialist for HIV treatment. At a one-week follow-up, skin discoloration remained, but the patient’s lesions continued to heal, and he was advised to continue acitretin and Daivobet.

## Discussion

This case presented a unique opportunity to observe dermatologic manifestations of numerous ailments at varying degrees in their course. Histopathology proved a clear diagnosis of psoriasis. Laboratory testing with a *Treponema pallidum* rapid plasma reagent (RPR) screening test and *Treponema pallidum* hemagglutination assay (TPHA) confirmed the diagnosis of syphilis and a rapid HIV antibody blood test provided the concurrent diagnosis. This case further demonstrated how syphilis, the great imitator, developed its notoriety. It is uncommon to see a myriad of infections progress to such an extent, especially in a relatively young patient at 17 years of age. Their complex interactions demonstrate the challenge of eliciting a dermatological diagnosis solely based on clinical signs and symptoms [4]. The provided images and clinical descriptions mapped very well with how a typical and uncomplicated case of psoriasis presents [5]. However, the lack of response to typical treatment clearly indicated that there were other factors at play. The immunosuppression due to HIV with a superimposed infection with *Treponema pallidum* demonstrated accelerated signs and symptoms. The pathogenicity of psoriasis and syphilis in HIV patients can prove to be paradoxical as therapies targeting T lymphocytes may improve the inflammatory effects of psoriasis while decreasing the CD4 and CD8 T-cell counts and exacerbating the immunodeficiency and superinfection [6]. This would warrant future monitoring for any lasting damage to avoid potential complications such as an aortic aneurysm or tabes dorsalis. Management of this disease triad may prove daunting as the clinical course becomes progressive and resistant to standard treatments. First-line treatment may include nonsteroidal anti-inflammatory drugs (NSAIDs), vitamin D analogs, vitamin A derivatives, and emollients [7]. We observed a vast improvement in the healing of the psoriatic lesions after two weeks of treatment with a combination of antibiotics, vitamin D, A, and E analogs, along with antihistamine and NSAIDs. A complicating factor in the treatment was the use of oriental medicine and treatment being delayed nine months after first contact with the healthcare facilities. There is no clear way of evaluating the effects these treatments may have had on the patient whether positive or negative. When the patient returned for treatment, he was already in the disease course. We recommend that care should be taken in the diagnosis of even seemingly uncomplicated cases by performing histopathology in addition to a thorough physical exam. In areas where endemic diseases are present, care should be taken to include them in the differential and learn to recognize their signs and symptoms in varying stages of presentation.

## Conclusions

The diagnosis of psoriasis is generally predicated on clinical signs and symptoms. Histopathology may be used as an adjunct to confirm the diagnosis and further establish a subtype. Upon initial presentation of a patient with advanced dermatological manifestations, care should be taken to rule out other diseases which may be concomitant. In developing regions of the world, endemic diseases should be included in the differential as a potential precipitating or contributing factor in the diagnosis. With skin manifestations, the timeline in which the lesions occur may clue a clinician into a disease course that may be atypical. A multisystem inflammatory disease, such as psoriasis, with such an accelerated onset and the extent of the spread of the lesion should raise the clinicians’ suspicion of other confounding factors. We recommend that care should be taken in the diagnosis of even seemingly uncomplicated cases by performing histopathology in addition to a thorough physical exam. In areas where endemic diseases are present, care should be taken to include them in the differential and learn to recognize their signs and symptoms in varying stages of presentation.
